The article "Reconstruction Algorithm-Based Computed Tomography Image Feature for Evaluating the Effect of Internal Administration and Medicated Bath of Liangxue Xiaoyin Decoction on Psoriasis Vulgaris" was published in 2022. Journal: Comput Math Methods Med.

# Reconstruction Algorithm-Based Computed Tomography Image Feature for Evaluating the Effect of Internal Administration and Medicated Bath of Liangxue Xiaoyin Decoction on Psoriasis Vulgaris

**DOI:** 10.1155/2022/7638507

**Published:** 2022-03-07

**Authors:** Fang Zhang, Jili Zou, Dandan Huang

**Affiliations:** ^1^Department of Chinese Medicine, Hubei College of Chinese Medicine, Jingzhou, 434020 Hubei, China; ^2^Department of Pharmacy, Wuhan Third Hospital, Wuhan, 430060 Hubei, China; ^3^Department of Chinese Medicine, Hubei Institute for Drug Control, Wuhan, 430075 Hubei, China

## Abstract

Skin computed tomography (CT) image based on improved marching cubes (MC) algorithm was explored to evaluate the therapeutic effect of internal administration of Liangxue Xiaoyin decoction combined with medicated bath in the treatment of psoriasis vulgaris. 712 patients with psoriasis vulgaris blood heat syndrome in hospital were recruited as the research object, which were randomly divided into observation group (TCM oral therapy combined with medicinal bath) and control group (TCM oral therapy), each with 356 cases. Psoriasis area and severity index (PASI), pruritus degree, and clinical treatment effect were compared. The results showed that the reconstruction time of median method was greatly shorter, and the algorithm efficiency was improved by 40.6290%. After treatment, the psoriasis area and severity index (PASI) score of the observation group was 5.61 ± 1.15, ΔPASI = (22.64 ± 2.15). ΔPASI% = 80.14%, which were greatly higher than the control group ((9.41 + 1.56) points, ΔPASI = (18.84 + 1.65) points, ΔPASI% = 66.69%) (*P* < 0.05). After treatment, the itching degree of the observation group was 3.03 ± 1.01 points, which was lower than that of the control group ((3.71 ± 1.06) points), and the itching degree of the observation group was greater than that of the control group, with substantial difference (*P* < 0.05). The total effective rate of observation group (88.76%) was higher than that of control group (71.07%) (*P* < 0.05). Therefore, skin CT image based on the improved MC algorithm can evaluate the therapeutic effect of internal administration of Liangxue Xiaoyin decoction combined with medicated bath in the treatment of psoriasis vulgaris. The internal administration of Liangxue Xiaoyin decoction combined with medicated bath had a good effect on the treatment of psoriasis vulgaris and was of certain clinical application value.

## 1. Introduction

Psoriasis is a common clinical skin disease. Psoriasis is a chronic inflammatory skin disease with a long onset time, which is easy to relapse and even cannot be completely cured [1]. The main clinical manifestation of the disease is that the plaque at the site of the disease is covered with multiple layers of red papules or silver-white phosphorous flakes, which are commonly found on the extension side of the limbs, back, and scalp, and even spread to the whole-body skin [2, 3]. According to the clinical manifestations of patients, psoriasis is classified into four types of pustular type, articular type, vulgaris type, and erythroderma type, among which the most common type is vulgaris type [4]. Traditional Chinese medicine classifies psoriasis vulgaris into blood heat, blood stasis, blood dryness, dampness heat, and dis-regulation of flushing, etc. through syndrome differentiation, among which blood heat syndrome is relatively common [5]. Currently, laser scanning confocal microscopy (LSCM) [6], also known as skin CT, is the main method for clinical examination of skin diseases. It is a noninvasive and high-resolution technique. Compared with traditional histopathological examination, this examination method is noninvasive, in situ, and in vivo detection, real-time, dynamic, repeatable, time-saving, and labor-saving, easy to store information, and has a wide scanning area. It is easy to find the characteristic changes of skin lesions and can be scanned by multiple points, so it is widely used in the development assessment and diagnosis and treatment of skin diseases [7]. The treatment of psoriasis is also a variety of methods, mainly classified into internal and external use of traditional Chinese medicine, western medicine, and external use. Liangxue Xiaoyin decoction is one of the prescriptions for oral treatment of Chinese medicine, which is used for the treatment of various psoriasis. As for external use, western medicine is used for external use to relieve patients' symptoms, but long-term use will cause side effects, and there is no radical cure, so Chinese medicine bath has been promoted. Both internal and external treatment in traditional Chinese medicine is symptomatic treatment based on syndrome differentiation, which has substantial effect [8].

The article "Reconstruction Algorithm-Based Computed Tomography Image Feature for Evaluating the Effect of Internal Administration and Medicated Bath of Liangxue Xiaoyin Decoction on Psoriasis Vulgaris" was published in 2022. Journal: Comput Math Methods Med.

To further enhance the performance of CT examination technology in clinical application and improve the accuracy of its examination, the reconstruction algorithm of medical image has been widely applied in the optimization of image examination images [9]. Various image reconstruction algorithms are used to optimize the display of medical images, including the reconstruction of 2D images into 3D images with intuitive stereoscopic effect. There are mainly two kinds of 3D reconstruction algorithms, namely, surface rendering and volume rendering. Marching cubes (MC) algorithm [10] belongs to one of the 3D reconstruction surface rendering algorithms, but MC itself may have some deficiencies.

To sum up, to improve the accuracy of research results, MC algorithm was improved and applied to evaluate the therapeutic effect of internal administration of Liangxue Xiaoyin decoction combined with medicinal bath in the treatment of psoriasis vulgaris, thereby providing more scientific and effective support for the treatment of psoriasis in traditional Chinese medicine and research support for the development of traditional Chinese medicine therapy.

## 2. Methods

### 2.1. Research Objects

A total of 712 patients with blood heat syndrome of psoriasis vulgaris admitted to hospital from January 2016 to March 2021 were selected as the study subjects. There were 412 male patients and 300 female patients, ranging in age from 18 to 65 years, with an average age of 38.56 ± 6.01 years. The distribution of lesions was 242 cases of mixed lesions, 30 cases of round skin lesions, 80 cases of chart lesions, 92 cases of disc lesions, and 268 cases of drip lesions. All patients were rolled into two groups with 356 cases in each group according to the random table method. The group of oral Chinese medicine therapy combined with bath therapy was set as the observation group, and the group of oral Chinese medicine therapy only was set as the control group. Moreover, CT images based on improved MC reconstruction algorithm were used to evaluate the therapeutic effect of the two groups. This study obtained the informed consent of patients and their families, who had signed the informed consent forms in strict accordance with relevant regulations. This study had been approved by ethics committee of the hospital.

Inclusion criteria are as follows: (a) patients who met the diagnostic criteria for traditional Chinese medicine psoriasis and the diagnostic criteria for advanced western psoriasis vulgaris in accordance with the *Consensus of Experts on Traditional Chinese medicine Treatment of Psoriasis of dermatology Branch* [11]; (b) patients who, after detailed explanation by the clinician, agreed to the treatment plan of this study and signed the relevant informed letter; (c) patients who did not use other drugs within one month before enrollment; (d) patients with complete clinical history.

Exclusion criteria are as follows: (a) patients with specific psoriasis; (b) patients with serious underlying diseases, such as tumors, cancers, and cardiopulmonary insufficiency; (c) pregnant or lactating women; (d) patients with mental and consciousness disorders; (e) patients who cannot make regular follow-up visits and cooperate with examinations.

### 2.2. Traditional MC Algorithm

The main principle of the traditional MC algorithm is as follows. First, the target space is divided by the volume element unit [12] (Figure 1), divided into multiple and detected one by one, and the voxel that intersects with the isosurface is found. Then, linear interpolation is used to calculate the intersection points with the isosurface, the normal vector is used to process the order of the isosurface, and finally, these surfaces are connected to complete the reconstruction of the 3D surface.

The article "Reconstruction Algorithm-Based Computed Tomography Image Feature for Evaluating the Effect of Internal Administration and Medicated Bath of Liangxue Xiaoyin Decoction on Psoriasis Vulgaris" was published in 2022. Journal: Comput Math Methods Med.

According to Figure 1, the sample value at point *C* is as follows.

(1) $$\begin{array}{c} C=\frac{x1-x}{\Delta x}\times \frac{y-y0}{\Delta y}\times \frac{z1-z}{\Delta z}\times D0+\frac{x1-x}{\Delta x}\times \frac{y1-y}{\Delta y}\times \frac{z1-z}{\Delta z}\times D1+\frac{x-x0}{\Delta x}\times \frac{y1-y}{\Delta y}\times \frac{z1-z}{\Delta z}\times D2+\frac{x-x0}{\Delta x}\times \frac{y-y0}{\Delta y}\times \frac{z1-z}{\Delta z}\times D3+\frac{x1-x}{\Delta x}\times \frac{y-y0}{\Delta y}\times \frac{z-z0}{\Delta z}\times D4+\frac{x1-x}{\Delta x}\times \frac{y1-y}{\Delta y}\times \frac{z-z0}{\Delta z}\times D5+\frac{x-x0}{\Delta x}\times \frac{y1-y}{\Delta y}\times \frac{z-z0}{\Delta z}\times D6+\frac{x-x0}{\Delta x}\times \frac{y-y0}{\Delta y}\times \frac{z-z0}{\Delta z}\times D7. \end{array}$$

After finishing, it is simplified as follows.

(2) $$\begin{array}{c} C\left(x,y,z\right)=b_{0}+b_{1}x+b_{2}y+b_{3}z+b_{4}xy+b_{5}yz+b_{6}zx+b_{7}xyz. \end{array}$$

In the above equation, *b*_0,1,2...7_ indicates constant values for the eight vertices. MC algorithm mainly finds the isosurface in the original data. It is assumed that the threshold value of this value is *Q*, then the isoface value is expressed as follows.

(3) $$\begin{array}{c} \left\{\left(x,y,z\right)\left|f\left(x,y,z\right)=Q\right.\right\}. \end{array}$$

Each *Q* point should be found to confirm the stitching order, which is confirmed by taking the normal vector of the triangular face. If the normal vector of each triangular surface is directly calculated and solved, the calculation will be large and complex. Therefore, the central difference method is often used for calculation, which is specifically expressed as follows.

(4) $$\begin{array}{c} q_{X}=\frac{f\left(X_{x+1},Y_{y},Z_{z}\right)-f\left(X_{x-1},Y_{y},Z_{z}\right)}{2\Delta X},\\ q_{Y}=\frac{f\left(X_{x},Y_{y+1},Z_{z}\right)-f\left(X_{x},Y_{y-1},Z_{z}\right)}{2\Delta Y},\\ q_{Z}=\frac{f\left(X_{x},Y_{y},Z_{z+1}\right)-f\left(X_{x},Y_{y},Z_{z-1}\right)}{2\Delta Z}. \end{array}$$

In the above equations, *q* is the order of elements in a volume.

### 2.3. Improved MC Algorithm

The traditional MC algorithm has the deficiency of low efficiency, so it is improved. First, data is preprocessed; CT images in digital imaging and communications in medicine (DICOM) [13] format are reconstructed. The DICOM standard CT image is converted into *bmp* format image, and the redundant information is removed, so as to speed up the processing. DICOM is an international standard for medical images and related information. CT images under this standard also contain other useless information, such as personal information, number, examination site, and shooting time. In 3D reconstruction, such information is not needed, so it is necessary to remove this information to reduce the data capacity, so the DICOM format is directly converted to *jpeg* or *bmp* format.

The article "Reconstruction Algorithm-Based Computed Tomography Image Feature for Evaluating the Effect of Internal Administration and Medicated Bath of Liangxue Xiaoyin Decoction on Psoriasis Vulgaris" was published in 2022. Journal: Comput Math Methods Med.

In the image interpolation processing, although the accuracy of linear interpolation is very high, the calculation method is relatively complex, so the median method is used instead of linear interpolation for image processing. The median method is a simpler interpolation method. For the coordinates of the intersection point, it simply needs to find the median of the corresponding coordinates of the edge.

It is supposed that the edge of the intersection is on the *x*-axis, then the coordinates of the intersection are as follows.

(5) $$\begin{array}{c} \left(X,Y,Z\right)=\left(x+\frac{1}{2},y,z\right). \end{array}$$

It is supposed that the edge of the intersection is on the *y*-axis, then the coordinates of the intersection are as follows.

(6) $$\begin{array}{c} \left(X,Y,Z\right)=\left(x,y+\frac{1}{2},z\right). \end{array}$$

It is supposed that the edge of the intersection is on the *z*-axis, then the coordinates of the intersection are as follows.

(7) $$\begin{array}{c} \left(X,Y,Z\right)=\left(x,y,z+\frac{1}{2}\right). \end{array}$$

With the rapid development of science and technology, CT slices are now only 2 mm to 5 mm apart. With the latest generation of imaging techniques, it is also possible to get sequences of smaller intervals. For such a small interval, the interpolation effect of using the median method is basically the same as that of linear interpolation. Therefore, the median method is used instead of linear interpolation method to shorten the calculation time and improve the efficiency.

### 2.4. Treatment Methods

The treatment method of control group was oral administration of Chinese medicine, and the Chinese medicine was Liangxue Xiaoyin decoction. The equation was 15 g each for buffalo horn, cortex moutan, Scubaaria baicalensis, Radix paeoniae paeoniae, Sophorae sophorae, rhizoma trichosanthiae, Radix daechedri, Radix sophorae, Radix sophorae, and Radix isatidis, 6 g each for gardenia and licorice, and 30 g of white flower hedyotis. To use it, the drugs were soaked in water for 4 h, then fried to 250 mL. There was one dose per day, half for morning and half for evening, for a four-week course of treatment, which requires three courses of treatment, that was, twelve weeks of treatment.

The article "Reconstruction Algorithm-Based Computed Tomography Image Feature for Evaluating the Effect of Internal Administration and Medicated Bath of Liangxue Xiaoyin Decoction on Psoriasis Vulgaris" was published in 2022. Journal: Comput Math Methods Med.

The treatment methods of the observation group were that the external therapy, namely, medicine bath therapy, was added based on the treatment methods of the control group. The composition of the medicine bath was the same as that of the traditional Chinese medicine for internal administration. 160 g of the medicine was added to 10 L water and soaked for about 5 h. Then, it was boiled with high heat and then simmered for 1 h. A small amount of warm water (i.e., up to the patient's hips while sitting in the tub) was added to the bath or tub. Then, the decoction was poured into the liquid, and the water temperature was controlled at about 40° for the bath. When the water temperature decreased, boiling water was added to adjust the temperature. A bath was taken once a day for 60 minutes each time. Continuous medication lasted for three courses, with two weeks as a course of treatment.

### 2.5. Skin CT Examination

Inspection tools were confocal laser scanning microscope and ultrasound gel. Scanning parameters were laser beam wavelength of 830 nm, power of 0-16 mW (adjustable), and lens of 30x water immersion objective lens. The horizontal resolution was 2 *μ*m (XY sequence), the vertical resolution was 1.6 *μ*m (Z sequence), and the epidermis and superficial dermis tissues within a depth of 200 *μ*m were scanned.

Operation procedure was as follows. First, a comfortable position was selected, the diseased position was exposed, photographed, and recorded, and the posture was maintained for 20-30 min. Then, a CT scan of the skin was performed.

First, a comfortable position was determined, and the disease part was exposed, photos were taken to record the disease position, and the posture was maintained for 20-30 minutes. Then, a CT scan of the skin was performed. Step 1: the skin CT operation interface was opened, and the patient's name, number, skin lesion site, and other information were input. Step 2: alcohol was used to clean the skin, excess scales were removed, and the skin surface was wetted. After the tissue ring was cleaned, the ultrasonic gel was squeezed into the skin lesion and connected with the skin CT probe. A certain pressure was maintained between the combined ring and the skin lesion. Step 3: the selected skin lesions were scanned and imaged. First, scanning was performed up and down to observe the imaging clarity of the interface. After obvious skin structure was visible on the display, the upper cuticle was marked as the vertical axis “0.” Scanning was performed up and down, and the thickness of the upper epidermis of the nipple at five different sites was measured and recorded. When obvious dermal papillary rings (basal and subcutaneous superficial dermal junction) were visible, scanning was performed on this horizontal plane. The diameters of five different dermal papillary rings were measured and recorded. Step 4: after the observation of typical skin lesions, normal skin within the adjacent range of 5 cm was selected for skin CT scan, and corresponding data were recorded.

The article "Reconstruction Algorithm-Based Computed Tomography Image Feature for Evaluating the Effect of Internal Administration and Medicated Bath of Liangxue Xiaoyin Decoction on Psoriasis Vulgaris" was published in 2022. Journal: Comput Math Methods Med.

### 2.6. Observation Indexes

#### 2.6.1. PASI Scoring Standards

Psoriasis area and severity index (PASI) [14] scoring standard is a method commonly used to assess the severity of psoriasis. The treatment effect was evaluated by comparing the area and severity of skin CT skin lesions before and after treatment. The specific CT skin lesion area scoring standard was presented in Figure 2.

Severity scoring standards were shown in Table 1.

After the lesion area and severity scores were determined, the final PASI score of the patient was determined according to the following equation, as presented in Figure 3.

According to Figure 3, the PASI score was calculated as follows.

(8) $$\begin{array}{c} \text{PASI score}=\left(E^{h}+I^{h}+D^{h}\right)*P^{h}*0.1+\left(E^{u}+I^{u}+D^{u}\right)*P^{u}*0.2+\left(E^{t}+I^{t}+D^{t}\right)*P^{t}*0.3+\left(E^{l}+I^{l}+D^{l}\right)*P^{l}*0.4. \end{array}$$

Therefore, if the PASI score before treatment was set as PASI ^before^ and the PASI score after treatment was set as PASI ^after^, the change value *Δ*PASI before and after treatment was expressed as follows.

(9) $$\begin{array}{c} \Delta \text{PASI}=\text{PAS}{\text{I}}^{\text{before}}‐\text{PAS}{\text{I}}^{\text{after}}. \end{array}$$

The change rate of lesion severity before and after treatment was *Δ*PASI%.

(10) $$\begin{array}{c} \Delta \text{PASI}\%=\frac{\left({\text{PASI}}^{\text{before}}‐\text{PAS}{\text{I}}^{\text{after}}\right)}{{\text{PASI}}^{\text{before}}}\times 100\%. \end{array}$$

#### 2.6.2. Itching Degree

The itching degree of patients before and after treatment was evaluated according to the *Criteria for Diagnosis and Curative effect of Dermatosis in Traditional Chinese Medicine* (Table 2).

#### 2.6.3. Evaluation of Treatment Effect

The therapeutic effect of the two groups of patients was evaluated according to the *Guiding Principles for Clinical Research of New Traditional Chinese Medicine*. The specific criteria were shown in Figure 4. 1 was recovery, 2 was effective, 3 was valid, and 4 was invalid. The total effective rate was the percentage of the sum of clinically cured, very effective, and effective.

The article "Reconstruction Algorithm-Based Computed Tomography Image Feature for Evaluating the Effect of Internal Administration and Medicated Bath of Liangxue Xiaoyin Decoction on Psoriasis Vulgaris" was published in 2022. Journal: Comput Math Methods Med.

### 2.7. Statistical Analysis

SPSS 22.0 statistical software was used. The measurement data were described with mean plus or minus standard deviation, and *t* test was performed. The counting data were described by percentage, and *χ*^2^ test was performed. *P* < 0.05 was considered statistically considerable differences.

## 3. Results

### 3.1. Algorithm Efficiency Comparison of Improved Interpolation Method

Figure 5 showed the comparison of reconstruction efficiency between linear interpolation and median method. When the number of triangles was the same as the number of vertices, the reconstruction time required by the linear interpolation method was 32.0023 seconds, while the reconstruction time required by the median method was only 19.0001 seconds. The time required for reconstruction was obviously shorter with the median method, and the algorithm efficiency was increased by 40.6290% (*P* < 0.05).  Figure 6 was a reconstruction effect diagram. The median method instead of linear interpolation was adopted, there was no substantial difference in reconstruction effect, and the surface of median method was smoother than linear interpolation.

### 3.2. Comparison of General Information of the Two Groups of Patients

Figure 7 showed the distribution of the gender ratio of the two groups of patients. The distribution of female patients in the two groups was 147 cases (49%) in the control group and 153 cases (51%) in the observation group (Figure 7(a)). The distribution of male patients in the two groups were 209 cases (50.73%) in the control group and 203 cases (49.27%) in the observation group (Figure 7(b)). There was no substantial difference in gender distribution between the two groups (*P* < 0.05).  Figure 8 showed the age distribution of the two groups of patients. The age range of all patients was classified into five stages of 18-30, 31-40, 41-50, 51-60, and 60 years old. Among them, the age distribution number corresponding to each age stage of the control group was 60 cases, 83 cases, 97 cases, 69 cases, and 47 cases, respectively (Figure 8(a)). The age the distribution number corresponding to each age stage of the observation group was 56 cases, 80 cases, 100 cases, 71 cases, and 49 cases, as presented in Figure 8(b). There was no substantial difference in the age distribution between the two groups (*P* < 0.05).  Figure 9 was a comparison of the distribution of skin lesions between the two groups of patients. Among them, there were 120 cases of mixed skin lesions in the control group, 14 cases of round lesions, 34 cases of pictorial lesions, 45 cases of discoid lesions, and 134 cases of spotted lesions. In the observation group, there were 122 cases of mixed lesions, 16 cases of round lesions, 46 cases of pictorial lesions, 47 cases of discoid lesions, and 134 cases of drip lesions. There was no substantial difference in the distribution of skin lesions between the two groups (*P* < 0.05), which suggested that the study was feasible.

The article "Reconstruction Algorithm-Based Computed Tomography Image Feature for Evaluating the Effect of Internal Administration and Medicated Bath of Liangxue Xiaoyin Decoction on Psoriasis Vulgaris" was published in 2022. Journal: Comput Math Methods Med.

### 3.3. PASI Score Results

Before treatment, the PASI score of the control group was 28.60 ± 2.21 points, and the observation group was 28.25 ± 2.05 points. After treatment, the PASI score of the control group was 9.41 ± 1.56 points, and that of the observation group was 5.61 ± 1.15 points; control group ΔPASI = (18.84 ± 1.65) points, ΔPASI% = 66.69%, and observation group ΔPASI = (22.64 ± 2.15) points, ΔPASI% = 80.14%. Through comparative analysis, the PASI scores of the two groups of patients before treatment were not greatly different (*P* > 0.05), and there were differences after treatment (*P* < 0.05). Moreover, through calculation, it was concluded that the *Δ*PASI and *Δ*PASI% of the observation group were higher than those of the control group, and the comparison was substantial (*P* < 0.05), as presented in Figure 10.  Figure 11 showed the skin lesions of the observation group before and after treatment. The area of the skin lesions was greatly reduced after treatment.

### 3.4. Degree of Itching and Curative Effect

In terms of the degree of pruritus, the degree of pruritus in the control group was 4.41 ± 1.36 points and that in the observation group was 4.27 ± 1.35 points before treatment, and there was no substantial difference (*P* > 0.05). After treatment, the degree of itching in the control group was 3.71 ± 1.06 points, and the observation group was 3.03 ± 1.01 points. The degree of pruritus change in the observation group was greater than that in the control group, and there was a substantial difference (*P* < 0.05) (Figure 12(a)). In terms of curative effect, 32 cases were cured in the control group, 158 cases were markedly effective, 63 cases were effective, and 103 cases were ineffective. In the observation group, 71 cases were cured, 213 cases were markedly effective, 32 cases were effective, and 40 cases were ineffective. The total effective rates of the two groups were 71.07% in the control group and 88.76% in the observation group, with substantial differences (*P* < 0.05), as presented in Figure 12(b).

## 4. Discussion

First, the MC algorithm was improved, and the detection results were analyzed. It was found that the effect of the median method was basically the same as that of the linear interpolation method, but the processing efficiency of the image was increased by 40.6290%. It suggested that the median method had good feasibility in the MC algorithm. This is basically consistent with the research results of a new 3D reconstruction algorithm for motion-blurred CT images [15]. The research by Ibáñez et al. [16] (2021) showed that the MC algorithm had a good application effect in imaging technology, which provided support for the credibility of this research. Then, the skin CT examination based on the improved MC 3D reconstruction algorithm was used to obtain the PASI score, to evaluate the therapeutic effect of internal administration of Liangxue Xiaoyin decoction combined with medicated bath in the treatment of psoriasis vulgaris. The PASI score (PASI = (5.61 ± 1.15) points, ΔPASI = (22.64 ± 2.15) points, ΔPASI% = 80.14%) of the observation group was greatly higher than that of the control group (PASI = (9.41 ± 1.56) points, ΔPASI = (18.84 ± 1.65) points, ΔPASI% = 66.69%) (*P* < 0.05). In addition, the total effective rate of the observation group (88.76%) was higher than that of the control group (71.07%) (*P* < 0.05). It was suggested that the therapeutic effect of oral administration of Chinese medicine combined with bath was better than that of single oral administration of the decoction, indicating that Chinese medicine therapy was of a good effect in the treatment of this disease. This was consistent with the findings of several research experts. Moreover, analysis of the clinical efficacy of treating psoriasis vulgaris with Chinese medicine bath showed that the combined treatment of patients with psoriasis vulgaris with Liangxue Xiaoyin decoction and traditional Chinese medicine bath can not only improve the therapeutic effect but also alleviate the disease of patients, which was recommended to promote [17]. In a series of studies on the treatment of moderate to severe psoriasis vulgaris by Chinese medicine combined with narrow-band UV-B irradiation, the patients with moderate and severe psoriasis were treated with the combination of Chinese medicine therapy and UV-B light therapy and achieved good efficacy [18]. In a systematic review and meta-analysis of the evidence and potential mechanisms of TCM treatment of psoriasis vulgaris, the results showed that TCM may be beneficial to lower PASI scores. Therefore, Chinese medicine may be an effective alternative therapy for the management of psoriasis vulgaris [19]. However, this study did not make a comparative analysis between Chinese medicine therapy and Western medicine therapy, which was a deficiency of this study. Most research results showed that the combined therapy of traditional Chinese medicine was better than the treatment effect of western medicine alone [20–23]. It may be related to the emphasis of traditional Chinese medicine therapy on treatment based on syndrome differentiation and the use of symptomatic drugs.

The article "Reconstruction Algorithm-Based Computed Tomography Image Feature for Evaluating the Effect of Internal Administration and Medicated Bath of Liangxue Xiaoyin Decoction on Psoriasis Vulgaris" was published in 2022. Journal: Comput Math Methods Med.

## 5. Conclusion

The skin CT image based on improved MC algorithm was used to evaluate the therapeutic effect of internal administration of Liangxue Xiaoyin decoction combined with medicated bath in the treatment of psoriasis vulgaris. The results showed that skin CT image based on the improved MC algorithm can evaluate the therapeutic effect of internal administration of Liangxue Xiaoyin decoction combined with medicated bath in the treatment of psoriasis vulgaris. The internal administration of Liangxue Xiaoyin decoction combined with medicated bath had a good effect on the treatment of psoriasis vulgaris and had certain clinical application value. However, there are still shortcomings in this study, such as failing to compare Chinese medicine with Western medicine. In the subsequent research, it needs to strengthen the comprehensiveness of the research comparison index. In summary, the traditional Chinese medicine bathing composition has a good therapeutic effect in treating patients with psoriasis vulgaris and is suitable for popularization and utilization.

## Figures and Tables

**Figure 1:** Unit diagram of body element.

**Figure 2:** Skin lesion area and score.

**Figure 3:** PASI scoring equation (*P*: skin lesion area score; *E*: spot color; *I*: degree of infiltration; *D*: scale performance; h: head; u: upper limbs; t: trunk; l: lower limbs).

**Figure 4:** Evaluation indicators of clinical treatment effect.

**Figure 5:** Comparison of reconstruction efficiency between linear interpolation and median method. (a) Reconstruction effect (A: number of triangles, B: number of vertices); (b) reconstruction time (L: linear interpolation, M: median method). “^∗^” indicated that the comparison was statistically significant (*P* < 0.05).

**Figure 6:** Comparison of reconstruction effects ((a) linear interpolation; (b) median method).

**Figure 7:** Comparison of gender distribution ((a) female; (b) male).

**Figure 8:** Age distribution ((a) control group; (b) observation group).

**Figure 9:** Distribution of skin lesions ((a) control group; (b) observation group; H: mixed shape; L: round shape; T: graph shape; P: disc shape; D: drip shape).

**Figure 10:** PASI scoring results. (a) PASI score before and after treatment; (b) *Δ*PASI; (c) *Δ*PASI%. “^∗^” indicated that the comparison was statistically significant (*P* < 0.05).

**Figure 11:** Skin lesions before and after treatment ((a–e) showed the appearance of skin lesions visible to the naked eye before treatment, (g–k) showed the skin lesions visible to the naked eye after treatment, (f) showed the appearance of skin CT skin lesions before treatment, and (l) showed the appearance of skin CT skin lesions after treatment).

The article "Reconstruction Algorithm-Based Computed Tomography Image Feature for Evaluating the Effect of Internal Administration and Medicated Bath of Liangxue Xiaoyin Decoction on Psoriasis Vulgaris" was published in 2022. Journal: Comput Math Methods Med.

**Figure 12:** Degree of itching and results of curative effect. (a) Degree of itching; (b) treatment effect. “^∗^” indicated that the comparison was statistically significant (*P* < 0.05).

**Table 1:** Skin lesion severity and score.

Score	0	1	2	3	4
Severity	No skin lesions	Mild	Moderate	Severe	Very severe
Specific manifestations					
Spot color	No spot	Light red	Red	Dark red	Black red
Degree of infiltration	Equal to normal skin	Slightly higher than normal skin	Moderate uplift	Obvious bulge	Very obvious bulge
Scale manifestations	No scales	Some were mainly fine scales	Most of them were flaky scales	Almost all scales were thick and layered	All scales were extremely thick and layered

**Table 2:** Itching score.

Score	Itching degree
0	No itching
2	Mild feeling, but did not affect normal life
4	Pruritus was paroxysomal and required medication, which had a certain impact on life
6	Severe itching, life was seriously affected

## Data Availability

The data used to support the findings of this study are available from the corresponding author upon request.
